The article "Effect of Intradialytic Change in Plasma Volume on Blood Pressure in Patients Undergoing Maintenance Hemodialysis" was published in 2010. Journal: J Lab Physicians.

# Effect of Intradialytic Change in Plasma Volume on Blood Pressure in Patients Undergoing Maintenance Hemodialysis

**DOI:** 10.4103/0974-2727.72151

**Published:** 2010

**Authors:** Ali-Reza Khalaj, Suzan Sanavi, Reza Afshar, Muhammad-Reza Rajabi

**Affiliations:** 1 Shahed University, Mustafa Khomeini Hospital, Tehran, Iran; University of Social Welfare and Rehabilitation Sciences, Akhavan Center, Tehran, Iran

**Keywords:** Blood pressure, body weight, hemodialysis, plasma volume

## Abstract

**Background:**

Hypervolemia is a common complication in patients on hemodialysis (HD). To determine the effect of volume change on blood pressure in HD population, this cohort was conducted.

**Materials and Methods:**

The study population was composed of 60 non-diabetic patients on maintenance HD, with mean age of 59.95±15.28 years. They were divided into hypertensive group A (*n*=26) and normotensive group B (*n*=34). Data were collected by a questionnaire. Pre and post-dialysis blood levels of urea, sodium, total protein, and hemoglobin were measured and intradialytic change of plasma volume were calculated. Data analyses were performed by the SPSS v.16.

**Results:**

Out of 60 patients, 58.3% were male and 41.7% female. Post-dialysis systolic blood pressure (SBP) and diastolic blood pressure (DBP) were significantly lower than pre-dialysis values in both groups (*P*=0.001, each). No correlation was found between intradialytic change in plasma volume or body weight and alterations of SBP or DBP during HD in the study groups (*P*>0.05, each). Intradialytic changes of body weight did not correlate to intradialytic changes of plasma volume (*P*=0.15).

**Conclusion:**

HD effectively reduces blood pressure and volume expansion, however, intradialytic changes of plasma volume and body weight do not influence on SBP and DBP.

## INTRODUCTION

Chronic renal failure (CRF) is a clinical syndrome due to various renal damages, which result in progressive and irreversible nephron loss. The most common causes of CRF include: diabetes mellitus, hypertension, glomerulonephritis, cystic disease, and interstitial nephritis.[1,2] Hemodialysis (HD) as a kidney-replacement therapy is the most common therapeutic modality in patients with end-stage renal disease (ESRD).[3] Apart from hemodialysis prescription, hypertension is a common complication in ESRD patients, so that nearly 85% of this population suffers from hypertension.[4] The causes of high blood pressure in hemodialysis patients are various including: sodium and fluid retention, rennin-angiotensin system over-activity, increased sympathetic activity and volume overloading.[5,6] Hypervolemia plays a major role in hypertensive patients on hemodialysis. Regardless of hypertension etiology, it is expected that removal of additional salt and water and restoration of dry body weight result in blood pressure normalization in about 60% of HD patients.[7,8] It is important to consider that the increase of extracellular volume may be insufficient to create edema and absence of edema does not rule out the presence of hypervolemia.[9] Control of volume status can normalize the blood pressure or facilitate blood pressure control in the majority of HD patients.[10] This study was conducted to determine the effect of plasma volume status on blood pressure in HD patients on maintenance HD.

The article "Effect of Intradialytic Change in Plasma Volume on Blood Pressure in Patients Undergoing Maintenance Hemodialysis" was published in 2010. Journal: J Lab Physicians.

## MATERIALS AND METHODS

This cohort study was performed on 60 non-diabetic patients, at the Mustafa Khomeini Hospital; Tehran; Iran, who were undergoing conventional (3 h for three times/weekly) maintenance HD. Indeed, patients with diabetes mellitus, symptomatic cardiac disease, severe illness, and history of hospitalization during prior 2 months were excluded. All participants were informed of study purposes and designed the consent forms. According to pre-dialysis blood pressure records during 2 months before the study, patients were assigned into group A (*n*=26), who were hypertensive (pre-dialysis blood pressure >140/90 mmHg) and received antihypertensive drugs and group B (*n*=34), who were normotensive without antihypertensive therapy. Data including demographic characteristics, underlying diseases, drugs, body weight and blood pressure records (pre- and post-hemodialysis), and biochemistry analyses were collected by a questionnaire. Pre- and post-dialysis (immediately at the end of dialysis) blood samples were drawn to obtain respective serum urea, sodium, total protein, and hemoglobin concentrations. Intradialytic change of plasma volume (∆ PV) was calculated by the *Leypoldt equation*[11] as follows:

$$∆\mathrm{PV}\;=\;[{\mathrm{PV}}_{\mathrm{pre}\;}-\;{\mathrm{PV}}_{\mathrm{post}}]\;÷\;{\mathrm{PV}}_{\mathrm{pre}\;}=\;[{\mathrm{TP}}_{\mathrm{post}}\;-\;{\mathrm{TP}}_{\mathrm{pre}}]\;÷\;{\mathrm{TP}}_{\mathrm{post}}$$

TP: total protein, pre: pre-dialysis, post: post-dialysis

In addition, urea clearance was calculated by logarithmic single pool *Kt/V (spKt/V*) equation according to the Daugirdas formula:[12]

spKt/V =(−In[ R − 0.008 × t ] + 4 − 3.5×R) × UF/W

Where *R* is the post–pre serum urea nitrogen (SUN) ratio, *t* is session length (in hours), UF is the volume of fluid removed during dialysis (in liters), and *W* is post dialysis body weight (in kilograms). In order to calculate *spKt/V*, the post-dialysis blood sample was drawn from arterial bloodline 20 s after dialysis session termination while the pump speed was reduced to 80 ml/min.

The article "Effect of Intradialytic Change in Plasma Volume on Blood Pressure in Patients Undergoing Maintenance Hemodialysis" was published in 2010. Journal: J Lab Physicians.

Data analyses were carried out, using the statistical software package SPSS, version 16. *P*-value <0.05 was considered statistically significant. The student’s *t*-test and Spearman’s test were used to detect significant differences between groups and correlations between variables.

## RESULTS

The study population consisted of 35 males (58.3%) and 25 females (41.7%), with mean age of 59.95 ± 15.28 years, who were undergoing maintenance HD (hemodialysis vintage = 6–34 months). Post-dialysis systolic blood pressure (SBP) and diastolic blood pressure (DBP) were significantly lower than pre-dialysis values in both groups (*P*=0.001, each). Table 1 shows details of blood pressure, body weight and plasma volume changes after HD and compares these values between two groups. However, there was no correlation between the intradialytic changes in plasma volume or body weight and pre- and post-dialysis SBP or DBP in both groups (*P*>0.05, each). In addition, no correlation was found between intradialytic change of body weight with intradialytic change in plasma volume (*P*=0.15). The Spearman test revealed only a positive correlation between the age and blood pressure (SBP and DBP) decrement (*P*=0.01 and *P*=0.026).

**Table 1:** Patients characteristics

Parameters	Group A (*n*=26)	Group B (*n*=34)	*P* value
Pre dialysis SBP (mmHg)	159.5±14.1	119.1±8.3	<0.001
Post dialysis SBP (mmHg)	139.6±13.8	110.5±8.5	<0.001
∆SBP (mmHg)	19±10.1	9±8.2	<0.001
Pre-dialysis DBP (mmHg)	91.3±7.5	80.2±7.2	<0.001
Post-dialysis DBP (mmHg)	82.1±7.4	70.2±7.3	<0.001
∆DBP (mmHg)	10±7.5	8±7.6	0.2
Pre-dialysis weight (kg)	68.6±10	63.7±10	0.03
Post-dialysis weight (kg)	65.5±10	61±10	0.03
∆BW (kg)	2.89±1.4	2.7±1.1	0.15
∆PV (%)	12.9±7. 3	12.5±6.6	0.51
*spKt/V*	1.09±0.3	1.09±0.3	

Values are Mean ± S.D.; ∆ = intradialytic change, BW = body weight, DBP = diastolic blood pressure, SBP = systolic blood pressure, PV = plasma volume

## DISCUSSION

In most patients with stable chronic renal disease (CRD), the total body contents of sodium (Na) and water are increased modestly which contributes to hypertension. When the glomerular filtration rate (GFR) falls to 5–10 ml/min, extracellular fluid volume (ECFV) expansion under these circumstances usually means that dialysis is indicated.[13] Patients with CRD also have impaired renal mechanisms for conserving Na and water. When an extrarenal cause for fluid loss is present, these patients are prone to volume depletion.[14] Hypertension is the most common complication of ESRD. Left ventricular hypertrophy and dilated cardiomyopathy due to prolonged hypertension and ECFV overload are among the most ominous risk factors for excess cardiovascular morbidity and mortality in patients with ESRD.[15] Absence of hypertension may signify the presence of a salt-wasting form of renal disease (medullary cystic disease, chronic tubulointerstitial disease, or papillary necrosis); ongoing antihypertensive therapy; volume depletion or reduced cardiac index. Since volume overload is the major cause of hypertension in uremia, the normotensive state can often be restored by appropriate use of salt restriction and ultrafiltration in the dialysis setting. Nevertheless, because of hyper-reninemia and other disturbances in renal vasoconstrictors and vasodilators, some patients remain hypertensive despite rigorous salt and water restriction and ultrafiltration.[16]

This study revealed that despite lower values of post-dialysis blood pressure, plasma volume, and body weight, compared to pre-dialysis values, there was no significant correlation between intradialytic volume status or body weight change and pre- or post-dialysis SBP and DBP. Such a result regarding the discrepancy between blood pressure and volume status has been reported previously.[17–20]

However, some researchers have shown the correlation between these variables. For instance, Lins and co-workers reported a positive correlation between SBP alteration and plasma volume change.[21] Leypoldt *et al*., and Ventura *et al*., have also got similar findings in this issue separately.[11,22] Furthermore, the HEMO study revealed that interdialytic weight gain correlated to high pre-dialysis blood pressure.[23] This finding had also been previously reported by Rahman *et al*.[24]

In our study, although eight patients in group B (normotensive) whose post-dialysis body weights were below 60 kg showed SBP reduction about 10 mmHg, however, we could not find significant correlation between intradialytic change in body weight and SBP. As mentioned previously, comparing to HEMO study, which had included patients with diabetes and cardiac disease, we excluded the categories that might have influences on refilling rate[25] and hemodynamic status. Our findings may be attributed to strict exclusion criteria of our study which finally led to selection of patients with high refilling rate of plasma volume (non-diabetic and appropriate cardiac function), so that the relationship between volume status, body weight and blood pressure was blunted. As a result, despite the differences in body weight (*P*=0.03) and blood pressure (P<0.001) between two study groups, the intradialytic plasma volume change was relatively similar in both groups Table 1. Indeed, the relationship between blood pressure and volume status in HD patients is not linear and various factors may affect this relation including dialysis dose and route (ultrafiltration), individual characteristics, refilling rate, cardiac function,[26] and vascular resistance.

The article "Effect of Intradialytic Change in Plasma Volume on Blood Pressure in Patients Undergoing Maintenance Hemodialysis" was published in 2010. Journal: J Lab Physicians.

Rocco and colleagues[23] reported that diabetes, old age, increased consumption of antihypertensive drugs and lower hematocrit values were associated with high SBP, whereas increased consumption of antihypertensive drugs and lower age were considered as DBP risk factors. In our study, among various variables including underlying disease, gender, age, hemoglobin, serum sodium, and serum urea, only age correlated with blood pressure levels.

As a whole, our findings are in agreement with previous researches and indicate that body weight change and plasma volume monitoring are not proper methods for evaluation of hydration status in HD patients. With regard to relation of SBP with intradialytic change of plasma volume in normotensive HD patients (which reflects absence of excessive extracellular fluid volume and high refilling rate) in some studies, it seems better to monitor combination changes of plasma volume and extracellular fluid volume, in HD population, to detect the influence of volume status on blood pressure.

## CONCLUSION

Despite, effective reduction of SBP, DBP, and plasma volume during hemodialysis, intradialytic changes of plasma volume and body weight do not influence on SBP and DBP. Many studies are proposed with consideration of other factors including residual renal function and extracellular fluid volume monitoring for evaluation of hydration status in hemodialysis patients.
